The article "Analysis of Bayesian posterior significance and effect size indices for the two-sample t-test to support reproducible medical research" was published in 2020. Journal: BMC Med Res Methodol.

# Analysis of Bayesian posterior significance and effect size indices for the two-sample t-test to support reproducible medical research

**DOI:** 10.1186/s12874-020-00968-2

**Published:** 2020-04-22

**Authors:** Riko Kelter

**Affiliations:** Department of Mathematics, University of Siegen, Walter-Flex-Str. 3, Siegen, Germany

**Keywords:** Bayesian significance and effect measures, Bayesian testing, Student’s t-test, Bayesian biostatistics

## Abstract

**Background:**

The replication crisis hit the medical sciences about a decade ago, but today still most of the flaws inherent in null hypothesis significance testing (NHST) have not been solved. While the drawbacks of *p*-values have been detailed in endless venues, for clinical research, only a few attractive alternatives have been proposed to replace *p*-values and NHST. Bayesian methods are one of them, and they are gaining increasing attention in medical research, as some of their advantages include the description of model parameters in terms of probability, as well as the incorporation of prior information in contrast to the frequentist framework. While Bayesian methods are not the only remedy to the situation, there is an increasing agreement that they are an essential way to avoid common misconceptions and false interpretation of study results. The requirements necessary for applying Bayesian statistics have transitioned from detailed programming knowledge into simple point-and-click programs like JASP. Still, the multitude of Bayesian significance and effect measures which contrast the gold standard of significance in medical research, the *p*-value, causes a lack of agreement on which measure to report.

**Methods:**

Therefore, in this paper, we conduct an extensive simulation study to compare common Bayesian significance and effect measures which can be obtained from a posterior distribution. In it, we analyse the behaviour of these measures for one of the most important statistical procedures in medical research and in particular clinical trials, the two-sample Student’s (and Welch’s) t-test.

**Results:**

The results show that some measures cannot state evidence for both the null and the alternative. While the different indices behave similarly regarding increasing sample size and noise, the prior modelling influences the obtained results and extreme priors allow for cherry-picking similar to p-hacking in the frequentist paradigm. The indices behave quite differently regarding their ability to control the type I error rates and regarding their ability to detect an existing effect.

**Conclusion:**

Based on the results, two of the commonly used indices can be recommended for more widespread use in clinical and biomedical research, as they improve the type I error control compared to the classic two-sample t-test and enjoy multiple other desirable properties.

## Background

In randomised clinical trials (RCT), the two-sample Student’s and Welch’s *t*-test is one of the most popular statistical procedures conducted. The goal often can be defined to test the efficacy of a new treatment or medication and investigate the size of an effect. Common settings use a treatment and control group, and the goal is to measure differences in a response variable like blood pressure. The gold standard in medical research for deciding if a new treatment or drug was more effective than the control treatment or drug is the *p*-value. The *p*-value states if the researcher can deem the observed difference significant, that means unlikely to have occurred under the assumption of the null hypothesis. The dominance of *p*-values when comparing two groups in medical (and other) research is overwhelming: Nuijten et al. [1] showed in a meta-analysis that of 258105 *p*-values reported in journals between 1985 and 2013, 26% belonged to a *t*-statistic, see also Wetzels et al. [2].

In its most restricted setting, the two-sample Student’s t-test assumes normally distributed data with identical variances, that is $Y_{1i}\sim \mathcal {N}(\mu _{1},\sigma ^{2}), Y_{2j}\sim \mathcal {N}(\mu _{2},\sigma ^{2})$ and tests the null hypothesis of no difference at all, that is *H*_0_:*μ*_2_=*μ*_1_, assuming equal sample sizes $i,j=1,...,n, n\in \mathbb {N}$. Removing the restriction for homoscedasticity – which is the assumption of identical variances $\sigma _{1}^{2} = \sigma _{2}^{2}$ in both groups – and the assumption of identical sample sizes *i*=*j*, the setting leads to the well known Behrens-Fisher-problem, which remains unsolved until today. The typical practice is to proceed with an approximative solution, known as *Welch’s two-sample t-test*. These approximative solutions are quite reliable, but as frequentist testing makes use of sampling statistics, which only allow rejecting the null hypothesis via the use of *p*-values, confirming any research hypothesis is not possible. The general procedure of null hypothesis significance testing (NHST), which uses sampling statistics to reject a null hypothesis via *p*-values makes formulating any reasonable research hypothesis complicated, as the research hypothesis first has to be rephrased in the form of a rejectable null hypothesis. In some cases, this is not possible at all, further limiting the usefulness of NHST in applied research. Countless papers have criticised the misuse and abuse of *p*-values in particular in medical research, and official statements of the American Statistical Association (ASA) in 2016 and 2019 by Wasserstein & Lazar [3] and Wasserstein et al. [4] make clear that tensions have not relaxed by now. The current practice shows that the *p*-value as a measure of significance is still widely used and resilient to the repeated criticism [5], while being prone to overestimating effects, stating effects if none exist in reality, and false interpretation by scientists [6]. This problem is especially observed in clinical research, see Ioannidis [7].

Among the proposed solutions to the problems of NHST is a shift to Bayesian statistics [4]. It is commonly agreed on that a more widespread use of Bayesian methods can at least partially improve the reliability in medical research on a statistical basis [8–10]. Recently, the development of Bayesian counterparts to frequently used statistical tests in medical and social science – including Student’s and Welch’s two-sample t-test – has opened up new possibilities for researchers: Open-source programs like JASP (https://jasp-stats.org) implement a broad spectrum of Bayesian methods and make them available to a wide range of researchers via a simple point-and-click user interface similar to SPSS.

Given the general recommendation of a shift towards the Bayesian paradigm, it is sensible to ask what benefits come with this shift. While NHST focusses on hypothesis testing via *p*-values and stating the significance of an observed effect, the Bayesian philosophy proceeds by the formulation of a statistical model, the inclusion of available prior information into the analysis, and the derivation of the posterior distribution of the parameters of interest, for example, the effect size in the setting of Student’s two-sample t-test. Employing the posterior *distribution* instead of point estimates, the Bayesian philosophy fosters estimation under uncertainty directly in contrast to NHST, which commonly uses point estimates like maximum likelihood estimates with confidence intervals, which are often interpreted wrong.

In NHST, testing for the significance of an effect is the standard approach, but the significance of an effect does not imply that the discovered relationship is also scientifically meaningful. It only means that the observed effect is unlikely to be observed under the assumption of the null hypothesis, no matter how large or small it is. Also, a non-significant result does not indicate that the null hypothesis is correct, and together these drawbacks of NHST can be seen as the reason why multiple measures of significance and magnitude of an effect based on the posterior distribution have been proposed in the Bayesian literature. In the Bayesian paradigm, inferences about the parameters of interest are drawn from the posterior distribution, and testing is optional. In practice, drawing conclusions from the posterior distribution is achieved by using different posterior indices. There are measures which state the significance of an effect, and measures which also gauge the size of it. Among them is the Bayes factor introduced by Jeffreys [11], the region of practical equivalence (ROPE) championed by Kruschke [12], the probability of direction (PD) as detailed in Makowski et al. [13], the MAP-based *p*-value proposed by Mills [14], and the Full Bayesian Significance Test (FBST) featuring the *e*-value, which was introduced by Pereira, Stern and Wechsler [15, 16]. The appropriateness of these indices is still debated in the literature, which makes it challenging to choose among the available indices because by now there is no explicit agreement on which index researchers should use to report the results of a Bayesian analysis [10, 17–19].

What is missing are specific investigations *which* of the available measures of significance and effect size are appropriate for a *specific* statistical method like the two-sample Student’s and Welch’s t-test. The results of such studies could guide scientists in the selection of an appropriate index to assess the result of a two-sample Student’s or Welch’s t-test performed in the analysis of clinical trial data. In order to provide such guidance, this paper investigates the behaviour of common Bayesian posterior indices for the presence and size of an effect in the setting of the two-sample Student’s and Welch’s t-test.

## Indices of significance and magnitude of an observed effect

In this section, we briefly review the existing Bayesian indices of significance and magnitude of an observed effect. Reviewing the most commonly used indices will serve as a firm understanding of the simulation study reported later in this paper, and also enhance a critical reflection on each of the indices.

### The Bayes factor (BF)

The oldest and still widely used index is the Bayes factor (BF). Bayesian hypothesis testing often is associated with the Bayes factor *BF*_01_, the predictive updating factor which measures the change in relative beliefs about both hypotheses *H*_0_ and *H*_1_ given the data *x*:

1 $$\begin{array}{*{20}l} \underbrace{\frac{\mathbb{P}(H_{0}|x)}{\mathbb{P}(H_{1}|x)}}_{\text{Posterior odds}} =\underbrace{\frac{p(x|H_{0})}{p(x|H_{1})}}_{BF_{01}(x)}\cdot \underbrace{\frac{\mathbb{P}(H_{0})}{\mathbb{P}(H_{1})}}_{\text{Prior odds}} \end{array} $$

The Bayes factor *BF*_01_ can be rewritten as the ratio of the two marginal likelihoods of both models, which is calculated by integrating out the respective model parameters according to the prior distribution of the parameters. Generally, the calculation of these marginals can be complex for non-trivial models. In the setting of the two-sample Student’s t-test, the Bayes factor is used for testing a null hypothesis *H*_0_:*δ*=0 of no effect against a one- or two-sided alternative *H*_1_:*δ*>0,*H*_1_:*δ*<0 or *H*_1_:*δ*≠0, where *δ*=(*μ*_1_−*μ*_2_)/*σ* is the effect size according to Cohen [20, p. 20], under the assumption of two independent samples and identical standard deviation *σ* in each group. An often lamented problem with Bayes factors as detailed in Kamary et al. [21] and Robert [17] is the dependence on the prior distributions assigned to the model parameters. Nevertheless, the Bayes factor has deep roots in Bayesian thinking and is one of the most widely used measures for hypothesis testing. Over the years, several authors including Jeffreys [11], Kass and Raftery [22] or Van Doorn et al. [23] have offered thresholds for interpreting different values of it. For example, according to Van Doorn et al. [23], a Bayes factor *BF*_10_>3 can be interpreted as moderate evidence for the alternative *H*_1_ relative to the null hypothesis *H*_0_, and a Bayes factor *BF*_10_>10 can be interpreted as strong evidence in the same way. Note that the Bayes factor *BF*_10_ can be obtained by inverting *BF*_01_ in equation (1), that is: *BF*_10_=*p*(*x*|*H*_1_)/*p*(*x*|*H*_0_)=1/*BF*_01_. So, if for example *BF*_01_=4 states moderate evidence for the null hypothesis *H*_0_:*δ*=0, then *BF*_10_=1/*BF*_01_ is obtained as 1/4 for the alternative hypothesis *H*_1_:*δ*≠0.

### The region of practical equivalence (ROPE)

The region of practical equivalence was championed by Kruschke [24], who stresses that such a region is often observed in different scientific domains under different names *“such as indifference zone, range of equivalence, equivalence margin, margin of noninferiority, smallest effect size of interest, and good-enough belt”* Kruschke [19, p. 272]. The essential idea is that in applied research, parameter values can often be termed practically equivalent if they lie in a given range. Starting from the posterior distribution of the parameter of interest, researchers should interpret values inside the region of practical equivalence (ROPE) as equivalent. For example, when conducting a clinical trial which compares the weight in kilograms of patients in two groups, one could define that the difference of means *μ*_2_−*μ*_1_ is practically equivalent to zero if it lies inside the ROPE [−1,1]. That means a difference of only one kilogram is interpreted as *practically equivalent to zero*. If the posterior distribution of *μ*_2_−*μ*_1_ now is entirely located inside the ROPE, the difference *μ*_2_−*μ*_1_ is interpreted as practically equivalent to zero a posteriori. On the other hand, if the total probability mass of the posterior distribution *μ*_2_−*μ*_1_ is located outside the ROPE, the null hypothesis *μ*_2_=*μ*_1_ of no difference can be rejected. The same procedure can be applied to any parameter, *θ* of interest. If the probability mass of the posterior lies partially inside and outside the ROPE, the situation is inconclusive.

There are two versions of the ROPE, one in which the 95% Highest-Posterior-Density-Interval (HPD) is used for the analysis (95% ROPE), and one in which the full posterior distribution is used (full ROPE). For the effect size *δ*, Kruschke [24] proposed to use [−0.1,0.1] as the ROPE for the null hypothesis *H*_0_:*δ*=0 of no effect, which is half of the effect size necessary for at least a small effect according to Cohen [20] (a small effect is defined as 0.2≤*δ*<0.5 or −0.5<*δ*≤−0.2 according to Cohen [20]).

### The probability of direction (PD)

The probability of direction is detailed in Makowski et al. [13] and varies between 50% and 100%. It is defined as the proportion of the posterior distribution of the parameter that is of the median’s sign. Therefore, if the posterior distribution assigns probability mass to both positive and negative parameter values, and the median is positive, it is the percentage of the posterior distributions probability mass located on the positive real numbers (0,*∞*).

### The MAP-based *p*-value

The MAP-based *p*-value was proposed by Mills [14] (see also Makowski et al. [13]), and can be related to the odds that a parameter has against the null hypothesis: It is defined as the ratio of the posterior density at the null value and the value of the posterior density at the maximum a posteriori (MAP) value, which is the equivalent of the mode for continuous probability distributions.

### The *e*-value and the full Bayesian significance test (FBST)

The Full Bayesian Significance Test (FBST) was originally developed by Pereira and Stern [15] and created under the assumption that a significance test of a sharp hypothesis had to be conducted. A sharp hypothesis refers to any submanifold of the parameter space of interest, see [16], which includes for example point hypotheses like *H*_0_:*δ*=0. Considering a standard parametric statistical model, where $\theta \in \Theta \subseteq \mathbb {R}^{p}$ is a (vector) parameter of interest, *p*(*x*|*θ*) is the likelihood function associated to the observed data *x*, and *p*(*θ*) is the prior distribution of *θ*, the posterior distribution *p*(*θ*|*x*) is proportional to the product of the likelihood and prior density:

$$\begin{array}{*{20}l} p(\theta |x) \propto p(x|\theta)p(\theta) \end{array} $$

A hypothesis *H* makes the statement that the parameter *θ* lies in the corresponding null set *Θ*_*H*_ then. Following [25] in notation, the Full Bayesian Significance Test (FBST) then defines two quantities: ev (*H*), which is the *e*-value supporting (or in favour of) the hypothesis *H*, and $\overline {\text {ev}}(H)$, the *e*-value against *H*, also called the *Bayesian evidence value against H*, see Pereira and Stern [15]. First, the posterior *surprise functions*(*θ*) and its maximum *s*^∗^ restricted to the null set *Θ*_*H*_ are denoted as

$$\begin{array}{*{20}l} s(\theta):=\frac{p(\theta|x)}{r(\theta)}, \hspace{1cm} s^{*}:=s(\theta^{*})=\sup\limits_{\theta \in \Theta_{H}}s(\theta) \end{array} $$

In the definition of the posterior surprise function *s*(*θ*), the denumerator *r*(*θ*) is a reference density. If the improper flat prior *r*(*θ*)∝1 is used, the surprise function becomes the posterior distribution *p*(*θ*|*x*). Otherwise, a noninformative prior distribution can be used as a reference density, see Stern [25]. The next step towards the *e*-value is to define

$$\begin{array}{*{20}l} T(\nu):=\{\theta \in \Theta|s(\theta)\leq \nu \}, \hspace{0.5cm} \bar{T}(\nu):=\Theta \setminus T(\nu) \end{array} $$

and $\overline {T}(s^{*})$ is then called the *tangential set to the hypothesis H*, which contains the points of the parameter space with higher surprise (relative to the reference density *r*(*θ*)) than any point in the null set *Θ*_*H*_. Integrating the posterior *p*(*θ*|*x*) over this set can be interpreted as the Bayesian evidence against *H*, the *e*-value $\overline {\text {ev}}(H)$:

$$\begin{array}{*{20}l} \overline{\text{ev}}(H):=\overline{W}(s^{*}), \hspace{0.5cm} W(\nu):=\int_{T(\nu)}p(\theta|x)d\theta \end{array} $$

Of course the *e*-value ev (*H*) supporting *H* is obtained as ev$(H):=1-\overline {\text {ev}}(H)$. In the above, *W*(*ν*) is called the cumulative surprise function, and $\overline {W}(\nu):=1-W(\nu)$. Therefore, large values of $\overline {\text {ev}}(H)$ indicate that the hypothesis *H* traverses low-density regions (or equivalently, that the alternative hypothesis traverses high-density regions) so that the *evidence against H is large*. The theoretical properties of the FBST and the *e*-value(s) have been detailed in Pereira and Stern [16] and Stern [25]. Here, we focus on the behaviour of the *e*-value $\overline {\text {ev}}(H)$ against *H*:*δ*=0 in the context of the Bayesian two-sample t-test. Note that one can use ev (*H*) to reject *H* if ev (*H*) is sufficiently small (or when $\overline {\text {ev}}(H)$ is large), but not to confirm *H*, which may be seen as a drawback of the FBST. Note also that there exist asymptotic arguments using the distribution of ev (*H*), which make it possible to obtain critical values based on this distribution to reject a hypothesis *H*, similar to *p*-values in NHST. In the simulation study reported later, we do not make use of any asymptotic argument and solely report the *e*-value $\overline {\text {ev}}(H)$ against *H*.

### Additional remarks

Makowski et al. [13] also proposed the Bayes factor versus ROPE index, which does not compare the point null hypothesis *H*_0_:*δ*=0 against an alternative *H*_1_:*δ*≠0 as the normal BF, but used a null *H*_0_:*δ*∈[−0.1,0.1] which is given by the ROPE and then tests against the alternative *H*_1_:*δ*∉[−0.1,0.1] which is the complement to the ROPE. While this approach is highly similar to the traditional ROPE and shows similar behaviour indeed [13], it will not be used here. Also, the frequentist *p*-value is used as a reference index, which is the probability under the null hypothesis, to obtain a result equal to or more extreme than the one observed for the statistical model used, see Wasserstein & Lazar [3].

Figures 1 and 2 show the different posterior Bayesian indices for significance and size of an effect for a Bayesian two-sample t-test. Group one was simulated as $\mathcal {N}(0.5,1)$ and group two as $\mathcal {N}(2,1)$ each with *n*=10 samples and the true effect size is *δ*=−1.5. The FBST is visualized in Fig. 1, where the left plot shows a Cauchy prior *C*(0,1) (dashed line) and the resulting posterior *p*(*δ*|*x*) (solid black line), which is obtained by the Bayesian two-sample t-test of Rouder et al. [26]. *s*^∗^ is computed as *s*(0)=0.1103 (indicated by the blue point) and the integral *W*(0) over the set *T*(0) is shown as the red area under the posterior. This area is ev (*H*), which is 0.0418 in this case. The blue area corresponds to the integral $\overline {W}(0)$ over the set $\overline {T}(0)$, which consists of all parameter values *δ* attaining a posterior density *p*(*δ*|*x*) larger than *p*(0)=0.1103, indicated by the horizontal dashed blue line. The value of this integral is the evidence against $H_{0}:\delta =0, \overline {\text {ev}}(H)=0.9582$, which advises the researcher to reject *H*_0_:*δ*=0 if a threshold of $\overline {\text {ev}}(H)>0.95$ is used for making a decision in light of the obtained evidence. The right plot in Fig. 1 shows the same situation, but now the reference prior *r*(*δ*) used in the surprise function has been changed from the improper flat prior *r*(*δ*)∝1 to the wide Cauchy prior *C*(0,1) actually used when conducting the Bayesian two-sample t-test of Rouder et al. [26]. Therefore, the surprise function values differ (see the scaling of the *y*-axis) and values of *p*(*δ*|*x*)/*p*(*δ*)>1 indicate that the posterior *p*(*δ*|*x*) assigns a larger probability to a given parameter value than the prior *p*(*δ*). This can be interpreted as the data having increased this parameters probability.

**Fig. 1:** Visualization of the Full Bayesian Significance Test. The *e*-value and FBST using a flat reference prior *r*(*δ*)∝1 (left) and wide Cauchy reference prior *C*(0,1) (right) against *H*_0_ for the Bayesian two-sample t-test; the blue area indicates the integral over the tangential set $\overline {T}(0)$ against *H*_0_:*δ*=0, which is the *e*-value $\overline {\text {ev}}$ against *H*_0_; the red area is the integral over *T*(0), which is the *e*-value ev (*H*) in favour of *H*_0_:*δ*=0

**Fig. 2:** Visualization of Bayesian posterior indices. Different Bayesian posterior indices for significance and size of an effect for a Bayesian two-sample t-test

The Bayes factor *BF*_10_ of *H*_0_:*δ*=0 against *H*_1_:*δ*≠0 is shown in the upper left plot of Fig. 2 and can be interpreted as the ratio of the prior density at the point-null value *δ*_0_=0 visualised as the grey lollipop and the posterior density at the point-null value *δ*_0_=0 visualised as the red lollipop. After observing the data, *H*_0_ becomes less probable, which is reflected in the Bayes factor of *BF*_10_=3.38. This magnitude indicates only moderate evidence for *H*_1_, which is due to the small sample size of *n*=10. Note that the Bayes factor *BF*_01_ can be obtained by inverting the ratio.

The MAP-based *p*-value is shown in the upper right plot and is defined as the ratio of the height of the posterior density at the null value *δ*_0_=0 and the MAP-value *δ*_*MAP*_, the maximum a posteriori parameter. As can be seen, the MAP estimate is near *δ*=−1, indicating a clear shift away from the null hypothesis. Still, the MAP-based *p*-value is given as *p*_*MAP*_=0.203, which is not significant.

The lower left plot visualises the 95% and full ROPE, where the ROPE is defined as [−0.1,0.1], following the recommendations of Kruschke [27]. 2.38*%* probability mass of the posterior distribution is located inside the ROPE when using the 95% ROPE and 3.00*%* is located inside the ROPE when using the full ROPE. In a test of practical equivalence, where the null is only rejected if the posterior is located entirely outside the ROPE, the null hypothesis *H*_0_ cannot be rejected based on the ROPE. Still, if an estimation-oriented perspective is used, avoiding the classical testing stance, the ROPE-analysis shows evidence for the alternative *H*_1_ for both the 95% and full ROPE.

The lower right plot in Fig. 2 shows the probability of direction (PD). It enjoys some desirable properties: First, it clearly shows that the effect is more likely to be of negative than positive sign, as 97.70*%* of the posterior is located on the negative real numbers. Also, the PD embraces estimation under uncertainty instead of hypothesis testing, in the same way as the ROPE does when avoiding an explicit testing stance. The posterior distribution can then be used in a second step to obtain, for example, the mean and standard deviation as estimates for the parameter. Still, hypothesis testing is also possible via rejecting the null *H*_0_:*δ*≥0 if at least 95% of the posterior of *δ* is located on the negative real axis.

## Methods

A simulation study was performed to analyse the behaviour of the different measures in the setting of Welch’s two-sample t-test. Pairs of data were simulated, consisting of two samples, one for each group, each normally distributed. Four settings were selected: In the first, no effect was present, and both groups were identically distributed as standard normal $\mathcal {N}(0,1)$. In the second, a small effect was present, and the first group was simulated as $\mathcal {N}(2.89,1.84)$ and the second as $\mathcal {N}(3.5,1.56)$, resulting in a true effect size of

2 $$\begin{array}{*{20}l} \delta=\frac{(2.89-3.5)}{\sqrt{((1.84^{2}+1.56^{2})/2)}}\approx -0.357 \end{array} $$

In the third simulation setting, a medium effect was present. The first group was simulated as $\mathcal {N}(254.08,2.36)$ and the second as $\mathcal {N}(255.84,3.04)$, resulting in a true effect size of

3 $$\begin{array}{*{20}l} \delta=\frac{(254.08-255.84)}{\sqrt{((2.36^{2}+3.04^{2})/2)}}\approx -0.646 \end{array} $$

The last setting used $\mathcal {N}(15.01,3.4)$ and $\mathcal {N}(19.91,5.8)$ distributions for the first and second group, yielding a true effect size of

4 $$\begin{array}{*{20}l} \delta=\frac{(15.01-19.91)}{\sqrt{((3.4^{2}+5.8^{2})/2)}}\approx -1.03 \end{array} $$

For each of the four effect size settings, 10,000 datasets following the corresponding group distributions as detailed above were simulated. This procedure was repeated for different samples sizes *n*, ranging from *n*=10 to *n*=100 in steps of size 10 to investigate the influence of sample size on the indices. In each case, the traditional *p*-value, the Bayes factor *BF*_10_, the ROPE 95%, the full ROPE, the probability of direction, the MAP-based *p*-value and the *e*-value $\overline {\text {ev}}(H_{0})$, that is the evidence against *H*_0_:*δ*=0 were computed. The Bayes factor was calculated as the Jeffreys-Zellner-Siow Bayes factor for the null hypothesis *H*_0_:*δ*=0 of no effect against the alternative *H*_1_:*δ*≠0, see Rouder et al. [26] and Gronau et al. [28]. More precisely, the calculated quantities are (1) the Bayes factor, a single number that quantifies the evidence for the presence or absence of an effect and (2) the posterior distribution, which quantifies the uncertainty about the size of the effect under the assumption *H*_1_:*δ*≠0 that it exists. This posterior distribution (2) of the effect size *δ* was then used to compute the 95% ROPE, the full ROPE, the PD and the MAP-based *p*-value as well as the *e*-value $\overline {\text {ev}}(H_{0})$. The traditional *p*-value was obtained via a two-sample Welch’s t-test.

The above procedure was conducted three times with the prior on the effect size *δ* set to three different hyperparameters to investigate the influence of the prior modelling: A noninformative Jeffrey’s prior was always put on the standard deviation of the normal population, while a Cauchy prior was placed on the standardised effect size. The Cauchy prior $C(0,\sqrt {2}/2)$ was used in the first setting, *C*(0,1) in the second and $C(0,\sqrt {2})$ in the third, corresponding to a medium, wide and ultrawide prior on the effect size *δ*. This way, the influence of the prior modelling on the resulting indices can be measured. To get more insights about the *e*-value $\overline {\text {ev}}(H_{0})$, for each prior setting $\overline {\text {ev}}(H_{0})$ was once computed using a flat improper reference density *r*(*δ*)∝1 (that is, the surprise function equals the posterior distribution), and once using the Cauchy prior assigned to *δ* as a reference density in the surprise function *s*(*δ*).

Finally, the above procedure was repeated for the fixed sample size *n*=30 to investigate the influence of noise. *n*=30 samples were simulated in each group to control for the influence of sample size and Gaussian noise $\mathcal {N}(0,\varepsilon)$ was added to the group data *x* and *y*, where *ε* was selected as *ε*=0.5 to *ε*=5 in steps of 0.5.

The percentage of significant results was computed for samples of increasing size *n* as the number of significant results divided by 10,000. This number is an estimate for the type I error probabilities of the indices, a quantity crucial for reproducible research [29]. Significant is defined here as follows: A Bayes factor *BF*_10_≥3. A posterior distribution using the 95% ROPE or full ROPE is significant when it is located completely outside the corresponding ROPE [−0.1,0.1] around *δ*=0. The MAP-based *p*-value is significant when *p*_*MAP*_<0.05. The *p*-value is significant when *p*<0.05. The PD is significant when *PD*=1 or *PD*=0, and the *e*-value is significant when $\overline {\text {ev}}(H)>0.95$ (no matter whether a flat reference density or the Cauchy reference density was used).

The statistical programming language R was used [30] for the simulations. The Bayes factor was computed via Gaussian quadrature in the R package BayesFactor [31], which was also used to obtain the posterior distribution of *δ* under the alternative *H*_1_ of an existing effect. The package bayestestR [32] was used to compute the 95% ROPE, full ROPE, PD and MAP-based *p*-value. The evidence $\overline {\text {ev}}$ against *H*_0_:*δ*=0 in the FBST was computed with the posterior Markov-Chain-Monte-Carlo draws of the posterior distribution of *δ* provided by the BayesFactor package [31]. These posterior draws were interpolated to construct a posterior density of *δ*, which was then integrated numerically over the tangential set of *H*_0_ as required for $\overline {\text {ev}}(H_{0})$. For more details, also about the random number generator seed, a commented replication script, which can reproduce all results and figures, is provided at the Open Science Foundation under https://osf.io/fbz4s/.

## Results

### Influence of sample size and prior modelling

Figure 3 shows the dependence of the Bayesian indices on sample size for four different effect sizes using the ultrawide prior $C(0,\sqrt {2})$. The four plots in each row show the succession of the results for no effect, a small effect, a medium effect and finally a large effect, while the x-axis shows increasing sample size *n*=10 to *n*=100 in each group in steps of 10.

**Fig. 3:** Influence of the sample size *n* on Bayesian significance and effect size indices for small, medium, large and no existing effects using an ultrawide prior $C(0,\sqrt {2})$ on the effect size *δ*

The left plot of the first row shows that the *p*-value is distributed uniformly under the null hypothesis *H*_0_:*δ*=0. If the alternative *H*_1_:*δ*≠0 is true, the three figures right beneath show that for increasing sample size *n*, the *p*-value becomes significant, where the necessary sample size for stating significance decreases with increasing actual effect size *δ*.

The second row shows the succession for the Bayes factor *BF*_10_. The left plot shows, that under the null hypothesis *H*_0_:*δ*=0 the Bayes factor correctly converges to zero (in contrast to the *p*-value). This property opens the possibility of confirming the null hypothesis, which is *not* possible via an ordinary *p*-value. The three figures right of this plot show the progression of the Bayes factor *BF*_10_ for increasing effect size. Here, the Bayes factor accumulates more and more evidence for the alternative *H*_1_:*δ*≠0 for small, medium and large effect sizes. For more substantial effect sizes, the Bayes factor requires a much smaller sample size to state evidence for the alternative. The plots are limited to a y-range of [0,100] (except for the first plot) for better visibility, as *BF*_10_ becomes very large quickly.

The third and fourth row shows the results for the 95% and full ROPE [−0.1,0.1] around the effect size *δ*=0. Under the null, in both cases, the percentage of the posterior’s probability mass inside the ROPE increases. As *δ*=0 under the null, for *n*→*∞*, the posterior will eventually concentrate completely inside the ROPE, but the necessary sample size can be considerable. From the figure, it becomes clear that for *n*=100, about 50% of the probability mass of the posterior is located inside the ROPE [−0.1,0.1] around *δ*=0. For increasing sample size *n*, this percentage will finally become 100%. Considering the 95% and full ROPE, even for small sample sizes like *n*=10 the majority of values shows that at least 10% of the posterior is located inside the ROPE so that hardly any false-positive statements are produced.

Under the alternative *H*_1_:*δ*≠0, both the 95% and full ROPE show that the percentage of the posterior located inside the ROPE [−0.1,0.1] of no effect converges to zero for increasing sample size *n*. For increasing effect size *δ*, the necessary sample size *n* needed to reject the null hypothesis *H*_0_ (based on an equivalence test or an estimation under uncertainty perspective as detailed by Kruschke [19]) becomes smaller.

The fifth row shows the results for the probability of direction (PD). Under the null hypothesis *H*_0_:*δ*=0, the PD is not uniformly distributed as was the case for *p*-values. The PD concentrates at about 70% here (see the scaling of the *y*-axis), which does not reflect the true effect size of *δ*=0, which should yield a PD near 50%. Still, under the alternative *H*_1_:*δ*≠0, the PD converges to 100% if sample sizes grow. The speed of convergence is faster for larger effect sizes *δ*≠0.

The MAP-based *p*-value shown in the sixth row shows a behaviour similar to the classic *p*-value. One difference is that under the null hypothesis *H*_0_, it is much larger on average than the traditional *p*-value. Still, this behaviour is robust to increasing sample size *n* and a correct interpretation of the MAP-based *p*-value only allows to state significance when *p*_*MAP*_ is smaller than a significance threshold. Interpreting large *p*_*MAP*_ as evidence for *H*_0_ is not allowed at all. Under the alternative *H*_1_, the behaviour is quite similar to the classic *p*-value: For increasing sample size *n*, the MAP-based *p*-value becomes significant, where the necessary sample size *n* for stating significance decreases with increasing effect size *δ*.

The evidence $\overline {\text {ev}}(H_{0})$ (in the following denoted as $\overline {\text {ev}}$) under the flat improper reference density *r*(*δ*)∝1 is shown in the seventh row and concentrates around *δ*=0.5 under the null hypothesis *H*_0_:*δ*=0. The reason for this can be seen in the fact that the posterior of *δ* concentrates for *n*→*∞* around *δ*=0 if *H*_0_:*δ*=0 is true, and the posterior density *p*(*δ*|*x*) also concentrates around *δ*=0 with slight fluctuations happening due to the randomness in simulation. The only thing that changes when increasing sample size *n* is thus the scaling of the *x*-axis of the posterior *p*(*δ*|*x*), so that $\overline {\text {ev}}$ is not influenced at all by increasing sample size. The support for *H*_0_ can easily be obtained by calculating ev$(H_{0})=1-\overline {\text {ev}}(H_{0})$, which in this case also concentrates around 0.5, instead of concentrating around 1. If on the other hand *H*_1_:*δ*≠0 is true, $\overline {\text {ev}}$ quickly signals evidence against *H*_0_ for increasing sample size *n* and increasing effect size *δ*, as shown by the three right-hand plots in the seventh row. When using the medium Cauchy prior $C(0,\sqrt {2}/2)$ instead of the improper reference density *r*(*δ*)∝1, the situation is similar, but the plots in the last row in Fig. 5 show that the evidence $\overline {\text {ev}}$ against *H*_0_ accumulate faster then if *H*_1_ is true.

Figure 4 shows the results of the simulation when using a wide prior *C*(0,1) instead of the ultrawide prior $C(0,\sqrt (2))$. The classic *p*-value is of course not affected at all from this prior change. The *BF*_10_ shown in the second row is slightly larger under the alternative *H*_1_:*δ*≠0, as the wide prior *C*(0,1) becomes more informative compared to the ultrawide prior $C(0,\sqrt {2})$. The probability mass located around *δ*=0 becomes more concentrated when using the wide *C*(0,1) prior instead of the ultrawide $C(0,\sqrt 2)$ prior, and therefore *BF*_10_ is increased (compare the boxplots in Figs. 3 and 4).

**Fig. 4:** Influence of the sample size *n* on Bayesian significance and effect size indices for small, medium, large and no existing effects using a wide prior *C*(0,1) on the effect size *δ*

**Fig. 5:** Influence of the sample size n on Bayesian significance and effect size indices for small, medium, large and no existing effects using a medium prior $C(0,\sqrt {2}/2)$ on the effect size *δ*

For the same reasons, the percentage of probability mass inside the 95% and full ROPE increases under the null *H*_0_:*δ*=0, as shown by the third and fourth row in Fig. 4. More prior mass around *δ*=0 due to the narrower *C*(0,1) prior on *δ* leads to more posterior mass inside the ROPE [−0.1,0.1] around *δ*=0. Under the alternative *H*_1_, the 95% and full ROPE suffer from this change, as shown in the boxplots for small, medium and large effects in rows three and four, which are shifted up slightly. The increase of probability mass near *δ*=0 draws the posterior towards *δ*=0, and it becomes harder for the posterior to concentrate outside of the ROPE. Nevertheless, for increasing sample size, the ROPEs finally reveal evidence for the alternative *H*_1_. Note that due to the concentration of probability mass around zero when using the *C*(0,1) prior, the boxplots of the ROPEs are shifted slightly up under the null hypothesis of no effect.

The same holds for the PD, which also needs a larger sample size now to achieve the same evidence for the alternative when an effect is present. No matter whether a small, medium or large effect size is present, all boxplots shift down slightly, indicating that less probability mass is strictly positive in the posteriors produced. The narrower prior distribution seems to shrink the complete posterior distribution towards smaller values, leading in turn to a smaller PD.

The MAP-based *p*-value is also influenced by the narrower prior: Due to the increased probability mass near *δ*=0, the MAP-estimate of *δ* shrinks towards *δ*=0. In combination with the larger value of the prior *C*(0,1) at the point-null value *δ*_0_=0 compared to the point-null value of the ultrawide prior $C(0,\sqrt {2})$, the ratio calculated for the MAP-based *p*-value decreases, leading to larger MAP-based *p*-values and slightly upshifted boxplots under the alternative *H*_1_.

The last two rows show $\overline {\text {ev}}$ under the improper reference density *r*(*δ*)∝1. Barely any change can be observed compared to the setting using the ultrawide prior $C(0,\sqrt {2})$, which is confirmed in the seventh row. Under the wide Cauchy prior reference density *r*(*δ*)=*C*(0,1), the evidence against *H*_0_:*δ*=0 again concentrates around $\overline {\text {ev}}=0.5$, indicating neither strong evidence against *H*_0_ nor support for *H*_0_. Compared to the ultrawide prior used in Fig. 3, under the alternative *H*_1_:*δ*≠0 the evidence $\overline {\text {ev}}$ against *H*_0_:*δ*=0 also barely changes. These results show that the *e*-value is quite robust against variations in the prior modelling.

Figure 5 shows the results when using a medium prior instead of a wide one. The classic *p*-value is again not affected from this prior, so the results are identical. In contrast to Figs. 3 and 4, the Bayes factor now accumulates evidence even faster, because the medium prior is even more informative than the wide and ultrawide one.

The 95% and full ROPE boxplots are shifted up even higher therefore under *H*_0_, showing that switching from the noninformative ultrawide and weakly informative wide prior to the medium prior yields larger percentages of the posterior distributions probability mass inside the ROPE under the null hypothesis *H*_0_ as even more probability mass concentrates around *δ*_0_=0 now. From a Bayesian perspective, the null hypothesis is thus faster confirmed. Under the alternative *H*_1_:*δ*≠0, the medium prior makes it now even harder for the 95% and full ROPE to reject the null hypothesis. This is again due to the fact that under the medium prior $C(0,\sqrt {2}/2)$ the prior allocates again more probability mass to values near *δ*_0_=0 than under the ultrawide $C(0,\sqrt {2})$ or wide Cauchy prior *C*(0,1). Therefore, the posterior shifts more slowly away from the ROPE [−0.1,0.1] of no effect, and therefore for the same sample size *n*, the posterior mass located inside the ROPE is larger when using the medium prior on *δ*. Still, for increasing sample size, this effect vanishes and even under the medium prior distribution, the concentration of posterior mass inside the ROPE converges to zero.

The same phenomenon holds for the PD and the MAP-based *p*-value. Here too, under the alternative the narrower prior on *δ* around zero makes it harder for the PD and MAP-based *p*-value to accumulate evidence for the alternative *H*_1_. For increasing sample size *n*, both the PD and the MAP-based *p*-value still finally reject the null hypothesis. For a fixed sample size *n*, the same is achieved faster under the ultrawide and wide prior, which have less prior probability mass near *δ*_0_=0.

Considering $\overline {\text {ev}}$ in the last two rows, under the improper reference density *r*(*δ*)∝1 again barely any changes can be observed compared to the setting using the ultrawide $C(0,\sqrt {2})$ or wide *C*(0,1) prior, which is confirmed in the seventh row of Fig. 5. Under the medium Cauchy prior reference density $r(\delta)=C(0,\sqrt {2}/2)$, the evidence against *H*_0_:*δ*=0 again concentrates around $\overline {\text {ev}}=0.5$, indicating neither strong evidence against *H*_0_ nor support for *H*_0_. Compared to the ultrawide and wide priors used in Figs. 3 and 4, under the alternative *H*_1_:*δ*≠0 the evidence $\overline {\text {ev}}$ against *H*_0_:*δ*=0 again is barely influenced by shifting to the medium Cauchy prior, showing strong robustness of the *e*-value against the prior modelling.

At this point, the results show that both the MAP-based *p*-value, the classic *p*-value and the *e*-value $\overline {\text {ev}}$ cannot state evidence for the null hypothesis in addition to being able to state evidence for the alternative. These measures can only reject the null hypothesis *H*_0_ and offer no possibility to confirm the null hypothesis. For practical research, this is limiting. Also, the PD stabilises at about 75%, which is the middle of its possible extremes, 50% and 100%. It would be desirable that the PD converges to 50% under the null *H*_0_:*δ*=0, to show that both a positive and negative effect are equally possible. Given the behaviour of the PD under the null, it seems that the PD favours the directed alternative *δ*>0 although the null *H*_0_:*δ*=0 is true. Under the alternative, *H*_1_:*δ*≠0, the PD as well as the *p*-value and MAP-based *p*-value behave as expected. Note that Pereira and Stern [15] created the *e*-value to test a sharp hypothesis *H*_0_, and rejection of *H*_0_ was the intended goal of the procedure. In contrast to the *p*-value and MAP-based *p*-value, the *e*-value enjoys a multitude of highly desirable properties like compliance with the likelihood principle, being a probability value derived from the posterior distribution, and possessing a version which is invariant to alternative parameterisations, see also [16]. Therefore, the *e*-value is preferable over the standard *p*-value and MAP-based *p*-value, also because of its robustness to the prior selection.

The Bayes factor *BF*_10_, the 95% and full ROPE have two desirable properties: Under the null, all three measures indicate evidence for *H*_0_:*δ*=0 while under the alternative *H*_1_:*δ*≠0, they indicate evidence for *H*_1_. It is somehow problematic while not astonishing that both constructs accumulate evidence faster under the null *H*_0_ using a medium prior, than when using a wide or ultrawide prior. Under the alternative, evidence for *H*_1_ accumulates faster when using a wide or ultrawide prior instead of a medium one. Thus, when using a medium prior, finding evidence for *H*_0_ is easier than finding evidence for *H*_1_ both with the BF and the ROPEs. Using a wide or ultrawide prior, finding evidence for *H*_1_ is easier than finding evidence for *H*_0_ with the BF and the ROPEs. Therefore, we recommend using the wide prior *C*(0,1), which places itself in the middle between these two extremes. Using a medium or ultrawide prior needs further justification, because otherwise, some kind of cherry-picking could happen by combining Bayes factors or ROPEs with a medium, wide or ultrawide prior depending on the goal of rejection or confirmation of the null hypothesis. Note that the *e*-value showed strong robustness to the prior selection. Therefore, if the rejection of a research hypothesis is the formulated goal of the scientific enterprise, the *e*-value based on the FBST procedure with the corresponding Cauchy prior as reference density in the surprise function may prevent such cherry-picking.

The take-away message regarding the prior modelling here is that the combination of prior and significance and effect size measure together can make it easier to find evidence for some hypotheses, which is problematic. Also, taking into account that the focus of research is to reveal relevant differences (clinically, in biomedical research for example), it is recommended to use at least *n*=100 patients in each group to ensure that also small effects can be detected reliably.

### Influence of noise

Figure 6 shows the results for the influence of noise on Bayesian indices of significance and effect size. As expected and shown in the first row, the influence of noise on the classic *p*-value under the null *H*_0_ is negligible. Under the alternative, the *p*-value gets disturbed more and more with increasing noise *ε*. The number of significant *p*-values reduces for increasing noise as shown by the boxplots, which are shifted upwards more and more when noise *ε* increases.

**Fig. 6:** Influence of noise *ε* on Bayesian significance and effect size indices for small, medium, large and no existing effects using a wide prior $C(0,\sqrt {2})$ on the effect size *δ* and sample size *n*=30 in each groups

The *BF*_10_ has the same problems: When the null hypothesis *H*_0_:*δ*=0 is true, the Bayes factor is not influenced much by noise. When on the other hand *H*_1_:*δ*≠0 is true, adding noise to the observations makes it more difficult for the Bayes factor to state evidence for the alternative *H*_1_:*δ*≠0. This behaviour is also revealed when comparing Figs. 3 and 6: The boxplots in the fourth plot of the second row in Fig. 3 show that the Bayes factor achieves higher values compared to the situation where noise is present, as shown in the fourth plot of the second row in Fig. 6.

The 95% ROPE and full ROPE also suffer from increasing noise. Under the null hypothesis, the noise does not influence the percentage of posterior mass inside the ROPE, but under the alternative *H*_1_ increasing noise *ε* causes increasing amounts of posterior mass to be located inside the ROPE. This behaviour makes it harder for the ROPE to signal evidence for the alternative *H*_1_:*δ*≠0.

The PD suffers from the same problem, as increasing noise causes the posterior to be more and more symmetric around *δ*_0_=0, indicated by the boxplots successively shifted down for increasing noise under *H*_1_.

The MAP-based *p*-value is also not influenced by noise under the null hypothesis *H*_0_, but the boxplots are shifted up under the alternative, indicating that increasing noise leads to larger *p*-values and less significant ones, which makes it harder for the MAP-based *p*-value to reject the null hypothesis in the presence of noise.

The *e*-value $\overline {\text {ev}}$ is also barely influenced by noise under the null hypothesis *H*_0_ both when used in combination with the flat reference density *r*(*δ*)∝1 and the wide Cauchy reference density *r*(*δ*)=*C*(0,1). Under the alternative, increasing noise makes it harder for $\overline {\text {ev}}$ to state evidence against *H*_0_ as shown in the last two rows of Fig. 6.

### Sensitivity and type I error rates

Table 1 shows Monte Carlo estimates for the type I error rates and the percentage of significant indices based on the results of the previous simulations. For increasing sample size *n*, the type I error rates were estimated as the number of significant indices divided by 10,000 when no effect was present.

**Table 1:** Percentage of significant Bayesian indices of significance and effect size for varying sample sizes for small, medium, large and no existing effects using a wide *C*(0,1) prior on the effect size *δ*

Index	*n*=10	*n*=20	*n*=30	*n*=40	*n*=50	*n*=60	*n*=70	*n*=80	*n*=90	*n*=100
No effect										
*p*-value	0.0483	0.0500	0.0552	0.0508	0.0507	0.0500	0.0491	0.0499	0.0520	0.0529
*BF*_10_	0.0221	0.0175	0.0192	0.0124	0.0137	0.0120	0.0104	0.0100	0.0100	0.0094
95% ROPE	0.0145	0.0159	0.0172	0.0127	0.0130	0.0107	0.0088	0.0083	0.0085	0.0069
Full ROPE	0.0002	0.0001	0.0000	0.0001	0.0000	0.0002	0.0000	0.0000	0.0000	0.0000
PD	0.0003	0.0003	0.0000	0.0004	0.0004	0.0006	0.0003	0.0003	0.0004	0.0002
MAP-*p*-value	0.0060	0.0075	0.0118	0.0096	0.0120	0.0111	0.0107	0.0107	0.0121	0.0117
$\overline {\text {ev}}$	0.0225	0.0273	0.0311	0.0342	0.0362	0.0383	0.0404	0.0386	0.0393	0.0391
$\overline {\text {ev}}$ with *C*(0,1)	0.0490	0.0470	0.0477	0.0459	0.0480	0.0471	0.0487	0.0458	0.0481	0.0474
Small effect										
*p*-value	0.1081	0.1990	0.2807	0.3457	0.4224	0.4890	0.5534	0.6149	0.6655	0.7092
*BF*_10_	0.0559	0.1045	0.1490	0.1835	0.2319	0.2682	0.3221	0.3648	0.4150	0.4562
95% ROPE	0.0433	0.0945	0.1423	0.1752	0.2238	0.2526	0.3014	0.3374	0.3831	0.4165
Full ROPE	0.0005	0.0012	0.0024	0.0047	0.0061	0.0107	0.0139	0.0186	0.0235	0.0289
PD	0.0010	0.0034	0.0090	0.0144	0.0265	0.0333	0.0538	0.0747	0.0953	0.1175
MAP-*p*-value	0.0222	0.0590	0.1082	0.1539	0.2137	0.2593	0.3219	0.3746	0.4369	0.4878
$\overline {\text {ev}}$	0.0671	0.1417	0.2252	0.2976	0.3720	0.4415	0.5171	0.5659	0.6175	0.6755
$\overline {\text {ev}}$ with *C*(0,1)	0.1164	0.1972	0.2763	0.3436	0.4180	0.4835	0.5527	0.5976	0.6459	0.7018
Medium Effect										
*p*-value	0.2762	0.5149	0.6930	0.8193	0.8899	0.9417	0.9717	0.9831	0.9907	0.9951
*BF*_10_	0.1709	0.3443	0.5013	0.6519	0.7439	0.8342	0.8928	0.9269	0.9561	0.9741
95% ROPE	0.1392	0.3247	0.4850	0.6389	0.7303	0.8197	0.8779	0.9165	0.9464	0.9685
Full ROPE	0.0017	0.0170	0.0382	0.0752	0.1282	0.1944	0.2769	0.3504	0.4386	0.5050
PD	0.0044	0.0320	0.0801	0.1635	0.2620	0.3830	0.4986	0.6010	0.6878	0.7606
MAP-*p*-value	0.0694	0.2431	0.4249	0.6039	0.7196	0.8256	0.8930	0.9317	0.9605	0.9779
$\overline {\text {ev}}$	0.1779	0.4373	0.6244	0.7698	0.8714	0.9256	0.9584	0.9752	0.9882	0.9951
$\overline {\text {ev}}$ with *C*(0,1)	0.2773	0.5227	0.6880	0.8083	0.8953	0.9376	0.9663	0.9807	0.9908	0.9960
Large Effect										
*p*-value	0.5824	0.8814	0.9746	0.9955	0.9987	1.0000	0.9999	1.0000	1.0000	1.0000
*BF*_10_	0.4438	0.7776	0.9254	0.9801	0.9937	0.9986	0.9999	0.9999	1.0000	1.0000
95% ROPE	0.3844	0.7584	0.9185	0.9787	0.9928	0.9984	0.9997	0.9999	1.0000	1.0000
Full ROPE	0.0182	0.1252	0.3133	0.5407	0.7192	0.8535	0.9259	0.9664	0.9851	0.9929
PD	0.0268	0.2052	0.4704	0.7217	0.8597	0.9450	0.9795	0.9933	0.9969	0.9997
MAP-*p*-value	0.0694	0.2431	0.4249	0.6039	0.7196	0.8256	0.8930	0.9317	0.9605	0.9779
$\overline {\text {ev}}$	0.4486	0.8367	0.9597	0.9927	0.9990	0.9996	1.0000	1.0000	1.0000	1.0000
$\overline {\text {ev}}$ with *C*(0,1)	0.5800	0.8862	0.9743	0.9945	0.9992	0.9998	1.0000	1.0000	1.0000	1.0000

Type I error rates and sensitivity of Bayesian posterior indices

In the cases where a small, medium or large effect was present, the percentage shows the number of significant measures divided by 10,000. Significant was defined as follows here: *p*<.05 for *p*-values, *BF*_10_≥3 for the Bayes factor, which equals moderate evidence according to Van Doorn et al. [23], a posterior which is located completely outside the 95% or full ROPE, and for the PD 100% of the posterior’s mass needed to be strictly positive or negative. The *e*-value $\overline {\text {ev}}$ against *H*_0_:*δ*=0 was required to be larger than 0.95, both when used with the improper reference density *r*(*δ*)∝1 and the wide Cauchy prior *r*(*δ*)=*C*(0,1) in the surprise function.

Figure 7 visualises the results: The left plot corresponds to the table row of no effect and shows the type I error rates of the indices. As shown in the figure, the classic *p*-value fluctuates around its nominal significance level of *α*=.05, although there is no effect present. In contrast, most Bayesian indices have lower type I error rates about half the size as the classic *p*-value. A comparison of the Bayesian posterior indices reveals three groups: The first group consists of the Bayes factor *BF*_10_, the 95% ROPE and the MAP-based *p*-value. These indices concentrate around a false-positive rate of about 1% for increasing sample size. Still, the Bayes factor and ROPE make more type I errors for small sample size, while the MAP-based *p*-value makes more for large sample sizes. The second group consists of the PD and the full ROPE, both of which make practically no type I error independent of the sample size *n*. This fact can be attributed to the quite conservative behaviour of both indices compared to the indices in group one. The third group consists of the *e*-value with improper or wide Cauchy prior, which achieves type I error rates slightly smaller than the traditional *p*-value, but more massive than the other Bayesian indices.

**Fig. 7:** Sensitivity of Bayesian significance and effect size indices for small, medium, large and no existing effects using a wide prior *C*(0,1) on the effect size *δ* and varying sample size *n*

The second plot corresponds to the small effect part of Table 1. Now the desired behaviour is that the indices detect the existing effect for the smallest possible sample size *n*. The classic *p*-value has the most liberate behaviour in stating that an effect is present, which reflects the often criticised fact that *p*-values overstate the significance of an effect compared to other indices of effect size and significance, see Wasserstein and Lazar [3]. The Bayesian indices signal evidence for the alternative more slowly than their frequentist counterparts, and again the three groups already discovered in the first plot reveal themselves here: The *BF*_10_, the 95% ROPE and the MAP-based *p*-value detect the small effect more often than the indices of the second group, which again includes the full ROPE and the PD. The third group consisting of the two versions of the *e*-value shows similar behaviour as the *p*-value: They signal the existence of an effect more quickly than their Bayesian competitors, which comes at the cost of increased type I errors as shown in the left plot previously.

The third and fourth plot correspond to the medium and large effect part of Table 1 and confirm the previous analysis. The *p*-value and *e*-value(s) state significance more often than every other index, but *BF*_10_, the 95% ROPE and the MAP-based *p*-value yield a similar behaviour for increasing effect size *δ* now. Also, from the succession of the PD and full ROPE, it becomes clear that the PD more often states the presence of an effect in contrast to the full ROPE, which is more conservative, even for increasing effect size. Still, for increasing sample size, these “slow“ indices eventually state the presence of the effect, too. Interestingly, the MAP-based *p*-value has a similar behaviour for large effect sizes as the full ROPE and PD, as shown in the right plot of Fig. 7. The behaviour of the *e*-value again shows substantial similarity to the behaviour of the *p*-value under the medium and large effect setting.

## Discussion

This paper studied the behaviour of common Bayesian significance and effect size indices for the setting of two-sample Welch’s t-test, which is often applied in the analysis of clinical trial data. To guide researchers in choosing an appropriate index when the Bayesian counterpart to Welch’s two-sample t-test as proposed by Rouder et al. [26] is used instead, an extensive simulation study analysed the influence of sample size *n*, the prior modelling and noise *ε*. Also, the type I error rates and sensitivities to detect an existing effect were studied.

The results show that one can split Bayesian significance and effect size indices into two categories: Indices which can state evidence for the null hypothesis *H*_0_:*δ*=0*and* the alternative *H*_1_:*δ*≠0, and indices which can only state evidence for the alternative. The first group consists of the Bayes factor, the 95% and full ROPE. The MAP-based *p*-value, the PD and the *e*-value belong to the second group, the MAP-based *p*-value and the *e*-value showing a similar behaviour as the classic *p*-value. Note that formally the *e*-value belongs to the first group, but the simulation results showed that stating evidence for the null hypothesis *H*_0_ is not achieved under the null hypothesis *H*_0_ by the *e*-value. On the other hand, the *e*-value showed the best performance compared to all other indices when *H*_1_ was true, and based on its other properties – for a review see Pereira, Stern and Wechsler [16] – it is preferable over the MAP-based *p*-value, PD and classic *p*-value. The PD suffers from the fact that under *H*_0_ it stabilizes at about 0.7, which is unintuitive and has to be interpreted as a tendency to favour evidence for the alternative when in fact the null hypothesis *H*_0_ is true, see Figs. 3, 4 and 5. Thus, when rejection of a null hypothesis is the goal, we recommend using the FBST and reporting the *e*-value based on the corresponding Cauchy prior as reference density in the surprise function. Also, the *e*-value is following the likelihood principle and is robust against the prior modelling, avoiding cherry-picking.

If the goal of the scientific enterprise is to confirm a research hypothesis, based on the results, the Bayes factor, the 95% ROPE or the full ROPE should be considered. All three indices show similar behaviour regarding increasing sample size *n*, and state both evidence for *H*_0_ and *H*_1_ depending on the presence of an effect.

The prior modelling showed that both the ultrawide and medium prior on *δ* could lead to cherry-picking by combining a selected index like a ROPE or BF with the prior: For example, choosing a medium prior when the goal is to confirm *H*_0_, evidence for *H*_0_ accumulates faster than when using a wide or ultrawide prior. If the goal is to find evidence for the alternative, evidence for *H*_1_ accumulates faster when using a wide or ultrawide prior instead of a medium one.

Therefore, we recommend using the wide prior *C*(0,1) when the goal is to confirm a hypothesis, as this choice places itself in the middle between the two other extremes and prevents cherry-picking in the case where no prior information is available.

The analysis of the influence of noise showed that all Bayesian indices suffered from increasing noise under *H*_1_ with no apparent patterns or regularities, or one of the indices being more robust to noise than the others.

The type I error rates, and the sensitivity to detect an existing effect revealed that all Bayesian indices should be preferred to the classic *p*-value, although the *e*-value showed only slightly reduced type I error rates compared to the traditional *p*-value. This result is essential, as the control of type I error rates is one of the most critical aspects in clinical trials, see McElreath [29] and Ioannidis [7]. The results showed further that the full ROPE and the PD achieve the best control of type I errors. As the PD cannot transparently state evidence for the null as shown previously, we recommend using the full ROPE to control type I errors in clinical trials.

While the Bayes factor, the MAP-based *p*-value, the *e*-value and the 95% ROPE are more sensitive and detect more effects when using the same sample size *n*, their type I error rate control is weaker.

## Conclusion

To guide researchers in the selection of an appropriate index for clinical trials, we recommend to use the full ROPE in general because of the following reasons: As the Bayes factor and 95% ROPE, the full ROPE can state evidence for both the null and the alternative hypothesis. The influence of sample size *n*, noise *ε* and prior modelling is similar for all three indices, but the type I error rate control is better for the full ROPE. The slightly weaker sensitivity to existing effects can be overcome by simply increasing the study sample size *n*, as shown in Fig. 7: For sample sizes of *n*=100, the sensitivity is nearly equal to the sensitivity of the Bayes factor and 95% ROPE when a large effect is present. When medium or small effects are present, larger sample sizes are required, but as often multiple hundreds of patients participate in clinical trials, the benefits of type I error control overshadow the higher costs incurred by increased sample size.^1^

Therefore, researchers and clinicians should benefit from using the full ROPE in the analysis of clinical trial data when conducting a two-sample Bayesian t-test through better type I error control and precise effect size estimation.

## Data Availability

The datasets generated and/or analysed during the current study as well as a full replication script to reproduce all results are available in the Open Science Framework (OSF) repository, https://osf.io/fbz4s/.

## Abbreviations

NHST: Null hypothesis significance testing
BF: Bayes factor
ROPE: Region of practical equivalence
PD: Probability of direction
MAP-based *p*-value: Maximum a posteriori based *p*-value
RCT: randomized clinical trial
ASA: American statistical association
JASP: Jeffreys awesome statistics package (software)
SPSS: Statistics package for the social sciences

## Footnotes

1 In the rare situation where the type I error rate is of less importance, we recommend to use the *e*-value instead, as it has the best sensitivity to detect an existing effect of all indices analysed, and is an attractive Bayesian replacement of the traditional *p*-value.
